This article has been retracted.

# Doppler Ultrasound under Image Denoising Algorithm in the Diagnosis and Treatment of Fetal Growth Restriction Using Aspirin Combined with Low-Molecular-Weight Heparin

**DOI:** 10.1155/2021/9697962

**Published:** 2021-10-16

**Authors:** Huiling Liu, Huiyuan Niu, Wenqiong Zeng

**Affiliations:** Department of Obstetrics, Huai'an Maternity and Child Care Hospital, Huaian 223001, Jiangsu, China

## Abstract

**Objective:**

This study explored the clinical application value of image denoising algorithm combined with Doppler ultrasound imaging in evaluation of aspirin combined with low-molecular-weight heparin (LMWH) on fetal growth restriction (FGR).

**Method:**

A two-stage image denoising by principal component analysis (PCA) with local pixel grouping (LPG-PCA) denoising algorithm was constructed in this study. Eighty FGR pregnant women were included in the study, and they were rolled into an experimental group (aspirin enteric-coated tablets + LMWH calcium injection) and a control group (LMWH calcium injection) according to the different treatment plans, with 40 cases in each group. All patients were performed with Doppler ultrasound imaging. The blood flow parameters (BFPs) were recorded and compared before and after the treatment in two groups, including power index (PI), resistance index (RI), high systolic blood flow velocity (S), high diastolic blood flow velocity (D), S/D value, and peak systolic velocity (PSV). In addition, the middle cerebral artery (MCA) BFPs, cerebral placental rate (CPR), amniotic fluid index (AFI) and perinatal outcome (PO) of the two groups were compared.

**Results:**

The total effective rate of treatment in group A (87.5%) was greatly higher than that in group B (62.5%), showing statistical difference (*P* < 0.05). The PI (0.72 ± 0.19), RI (0.57 ± 0.17), and S/D values (2.26 ± 0.43) in group A were dramatically lower than those in group B, which were 0.92 ± 0.21, 0.75 ± 0.14, and 2.64 ± 0.45, respectively (*P* < 0.05), and the AFI was higher (13.71 ± 2.2 cm vs 11.38 ± 2.16 cm) (*P* < 0.05). The Apgar score (9.17 ± 0.26), weight (3.57 ± 1.08), and gestational age (38.85 ± 2.50) of group A were all higher in contrast to those of group B, which were 7.33 ± 0.25, 2.61 ± 1.13, and 36.18 ± 2.25, respectively (*P* < 0.05). In addition, the fetal double parietal diameter (2.4 ± 0.9 mm), femur diameter (2.2 ± 0.6 mm), head circumference (1.2 ± 0.4 mm), abdominal circumference (1.3 ± 0.7 mm), and uterine height (0.8 ± 0.3 mm) in group A were obviously superior to those in group B, which were 1.8 ± 0.4 mm, 1.7 ± 0.5 mm, 0.8 ± 0.2 mm, 0.9 ± 0.4 mm, and 0.4 ± 0.6 mm, respectively, showing statistically observable differences (*P* < 0.05).

**Conclusion:**

Doppler ultrasound based on image denoising algorithm can accurately evaluate the effect of aspirin combined with LMWH on the improvement of FGR and showed good application value.

## 1. Introduction

Fetal growth restriction (FGR) is defined as a child whose fetus is unable to achieve its intended growth potential and is small for its gestational age (birth weight is less than the 10th percentile below the weight of the same age), and it is also a relatively common disease in obstetrics [1]. In addition to affecting the growth and development of the fetus, it can also induce complications such as premature birth, cerebral palsy, fetal asphyxia, and even death [2]. Studies have found that the blood of FGR pregnant women is in a state of hypercoagulability [3,4], so improving the hypercoagulable state of pregnant women and placental blood perfusion is the key to the treatment of FGR [5]. Therefore, timely and effective treatment of FGR is the key to improving the prognosis of perinatal infants. Low-molecular-weight heparin (LMWH) has a certain effect in the treatment of FGR. It has effects on improving uterine placental blood circulation, reducing blood viscosity, and enhancing placental blood supply [6,7], but monotherapy is still insufficient. Aspirin is a common antipyretic and analgesic drug. It was firstly used for antipyretic and analgesic, and now it is mainly used as an antiplatelet aggregation drug to prevent cardiovascular and cerebrovascular diseases. Related studies have found that aspirin can improve placental function, improve clinical pregnancy rate, and reduce the incidence of recurrent miscarriage [8].

Clinical examination methods for FGR mainly include medical history collection and physical examination, Doppler ultrasound, amniocentesis, and chromosome examination. Among them, medical history collection and physical examination are to look for FGR-related diseases to indirectly assess the occurrence of FGR. Amniocentesis can perform a specific amniotic membrane virus DNA test to determine whether the fetus has intrauterine growth restriction. Chromosome examination can be performed when FRG is early-onset and well-proportioned (midterm pregnancy), severe (fetal weight is less than the 3rd percentile), or accompanied by polyhydramnios. To adopt the most beneficial treatment plan for pregnant women and fetuses, it needs to be based on comprehensive and detailed ultrasound examination. At present, the most commonly used clinically is color Doppler ultrasound, which is a medical device suitable for examination and diagnosis of various parts of the body, especially the abdomen, obstetrics, and gynecology. It refers to, in the case of two-dimensional echocardiographic positioning, using the principle of Doppler and a series of electronic technologies to display the spectrogram of the blood flow in the body in real time, and it has the advantages of noninvasiveness and high sensitivity [9]. It plays an important role in evaluating the growth status of the fetus in the uterus and detecting hemodynamics. However, during color Doppler imaging, some white or black points often appear randomly in the image, which may result from the noise caused by the interference of the image signal, reducing the signal-to-noise ratio of the image and cause artifacts [10], so that error information is obtained, which adds unnecessary burden to clinical work. Therefore, it is necessary to effectively denoise Doppler ultrasound images.

Principal component analysis (PCA) is a statistical method that transforms potentially correlated variables into linearly uncorrelated variables through orthogonal transformation. The transformed variables are the principal components. K. Pearson is the first introduced nonrandom variable, which was generalized to the random vectors by H. Hotelling. At the beginning of the twenty-first century, researchers have applied PCA to image denoising, which is more effective and simpler than traditional methods [11]. However, there are also some problems such as noise remaining, so some scholars have upgraded the PCA method. At this time, the two-stage image denoising by principal component analysis with local pixel grouping (LPG-PCA) was proposed, which not only can handle the residual noise well and improve the signal-to-noise ratio but also can retain the image data information to the maximum.

This study explored the therapeutic effect of aspirin combined with LMWH on 80 FGR pregnant women under the color Doppler ultrasound evaluation based on the LPG-PCA image denoising algorithm, so as to analyze its effect on the clinical efficacy of FGR.

## 2. Research Methods

### 2.1. Research Objects

Eighty cases of FGR pregnant women, aged 24–43 years, who presented to the hospital from March 2019 to August 2020 for disease examination and treatment, were selected as research objects. They were rolled into an experimental group (aspirin enteric-coated tablets + LMWH calcium injection) and a control group (LMWH calcium injection) according to the different treatment plans, with 40 cases in each group. The medical ethics committee of our hospital approved the study, and the study objective was explained to the family members of the patients and children and they signed informed consent forms.

The inclusion criteria were defined as follows: patients with FGR confirmed by ultrasound examination; patients with complete clinical data; patients who were singleton pregnancy; patients who signed the informed consents.

The exclusion criteria were defined as follows: patients with severe complications during pregnancy such as diabetes and hypertension; patients who suffered from fetal malformations or chromosomal abnormalities; patients who combined with severe organic diseases; patients who were allergic to the drug in this study.

### 2.2. Treatment Schemes

Patients in group B received LMWH calcium injection (Shenzhen Saibaoer Biopharmaceutical Co., Ltd.), with once a day, 25,000 IU each time, and subcutaneous injection. One course of treatment was calculated as one week of continuous treatment, and the next course of treatment was continued for one week. The continuous treatment should last for three courses. Patients in group A were treated with aspirin enteric-coated tablets (Bayer Healthcare Co., Ltd.), once a day, 25 mg each time, orally, for three consecutive courses.

### 2.3. Doppler Ultrasonic Examination

The ACUSON Juniper whole body application color Doppler ultrasound diagnostic apparatus (SIEMENS Company, Germany) was adopted for examination, with the convex array probe and the frequency of 3.0–5.0 MHz. After the pregnant woman drunk water to fill her bladder, she lied on her back on the examination bed and breathed evenly. An experienced professional imaging physician would conduct a comprehensive scan of the fetus, check the status of various structures and appendages, and measure the growth of the fetus in various sections according to the guidelines of the International Society of Obstetrics and Gynecology and Ultrasound.

### 2.4. Observation Indicators

To evaluate the effects of the two groups, color Doppler ultrasound was adopted to detect the UA blood flow and amniotic fluid before and after treatment, and the umbilical artery (UA) blood flow parameters (BFPs) (power index (PI), resistance index (RI), high systolic blood flow velocity (S), high diastolic blood flow velocity (D), and S/D value), middle cerebral artery (MCA) BFPs (PI, RI, S, D, and S/D value), amniotic fluid index (AFI), and fetal cerebral placental rate (CPR) were recorded and compared. Before treatment and after a course of treatment, the pregnant women's uterine height and abdominal circumference growth were measured. The fetal growth (fetal head double parietal diameter, femur length, head circumference, and abdominal circumference) was detected using the color Doppler ultrasound. In addition, the maternal and infant outcomes were recorded and compared, including premature abruption, fetal distress, oligohydramnios, and postpartum hemorrhage for parturient and Apgar score, weight, gestational age, premature birth, and full-term infants for newborn.

### 2.5. Evaluation Criteria

FGR efficacy criteria were as follows. If the growth rate of pregnant women's uterine height and abdominal circumference had been greatly accelerated, the biparietal diameter increased by ≥ 1.4 mm per week, and there were no neonatal complications. It could be determined as “markedly effective.” If the uterine height and abdominal circumference of pregnant women had increased but not obviously, the double parietal diameter increases by 1.4–2.0 mm every two weeks, and there were no neonatal complications. This was defined as “effective.” If the uterine height and abdominal circumference of the pregnant woman did not increase, the double parietal diameter did not increase dramatically, and neonatal complications occurred. This was deemed as “ineffective.” The total effective rate = (the number of patients with effective effect + the number of patients with markedly effective effect)/total number of cases × 100%.

### 2.6. Image Denoising Algorithm

A certain pixel in the image and the *A∗A* topological interval were considered as a vector, which was represented by *x*_*f*_=[*x*_1_^*f*^,…,*x*_*n*_^*f*^]^*Q*^, *f*=[*f*_1_,…,*f*_*n*_]^*Q*^, and *n*=*A*^2^. All elements in the topological interval set were also regarded as vectors. The vector of an ultrasound image with noise was expressed in the following form:

(1) $$\begin{array}{c} x_{f}=x+f. \end{array}$$

The sample matrix *u* × *v* of *X*_*f*_ can be expressed in the form of *X*_*f*_=[(*X*_1_^*f*^)^*Q*^,…,(*X*_*n*_^*f*^)^*Q*^]^*Q*^ and *X*_*f*_=*X*+*F*. The average value of *x*_*a*_^*f*^ was expressed as *p*_*a*_=1/*v*∑_*i*=1_^*v*^*X*_*a*_^*f*^(*i*). *X*_*f*_ can be expressed in the form of ${\bar{X}}_{a}^{f}=X_{a}^{f}-p_{a}$ after decentralization, and the decentralized form without noise can be expressed as ${\bar{X}}_{a}=X_{a}-p_{a}$. Then, the two conformed to the following equation:

(2) $$\begin{array}{c} {\bar{X}}_{f}=\bar{X}+F. \end{array}$$

The expression of the covariance matrix of ${\bar{X}}_{f}$ was as follows:

(3) $$\begin{array}{c} C_{{\bar{X}}_{f}}=\frac{1}{v}{\bar{X}}_{f}{\bar{X}}_{f}^{Q}\approx \frac{1}{v}\left({\bar{XX}}^{Q}+{\bar{FF}}^{Q}\right)=C_{\bar{X}}+C_{f}. \end{array}$$

There was no correlation between *v*_*i*_ and *v*_*j*_, so *C*_*f*_=*ϕ*^2^*R* can be changed to the following form:

(4) $$\begin{array}{c} C_{{\bar{X}}_{f}}=C_{\bar{X}}+C_{f}=P_{\bar{X}}\Lambda \bar{X}\Lambda P_{\bar{X}}^{Q}+P_{\bar{X}}\left(\phi^{2}R\right)P_{\bar{X}}^{Q}=P_{\bar{X}}\left(\Lambda_{\bar{X}}+\phi^{2}R\right)P_{\bar{X}}^{Q}=P_{\bar{X}}\Lambda {\bar{X}}_{f}\Lambda P_{\bar{X}}^{Q}. \end{array}$$

The previously mentioned equation showed that $C_{{\bar{X}}_{f}}$ and $C_{\bar{X}}$ shared the same eigenvector matrix $P_{\bar{X}}$, the expression of which after conversion was as follows:

(5) $$\begin{array}{c} S_{\bar{X}}=P_{\bar{X}}^{Q}. \end{array}$$

The following equation could be obtained by conversing the ${\bar{X}}_{f}$:

(6) $$\begin{array}{c} {\bar{Y}}_{f}=S_{\bar{X}}{\bar{X}}_{f}. \end{array}$$

Then, it could only process ${\bar{Y}}_{f}$ to get the noise-free $\bar{X}$. By analogy, the previously mentioned operations were performed on each pixel value in the image, and then the denoised ultrasound image could be obtained (Figure 1.

### 2.7. Statistical Analysis

SPSS 20.0 was used for data processing, and the count data used the *χ*^2^ test; $\bar{x}\pm s$ represented the measurement data, and the *t*-test was used. *P* < 0.05 meant the difference was statistically significant.

## 3. Results

### 3.1. Comparison on Basic Data of Patients in Two Groups

Compared with group B, the data of group A patients were not statistically different (*P* > 0.05), as given in Table 1.

### 3.2. Clinical Efficacy

The total effective rate in group A (87.5%) was obviously higher than that of group B (62.5%), and the difference was statistically significant (*P* < 0.05), as shown in Table 2.

### 3.3. Fetal UA BFPs and AFI before and after Treatment

Color Doppler ultrasound based on denoising algorithm (Table 3) showed that there was no great difference between the two groups of fetal PI, RI, S/D, PSV, and AFI before treatment (*P* > 0.05); after treatment, the PI (0.72 ± 0.19), RI (0.57 ± 0.17) and S/D (2.26 ± 0.43) in group A were much lower than the previously mentioned indicators in group B, which were 0.92 ± 0.21, 0.75 ± 0.14, and 2.64 ± 0.45, respectively (*P* < 0.05). AFI (13.71 ± 2.2) was much higher than group B (11.38 ± 2.16) (*P* < 0.05), but there was no marked difference in the PSV between two groups (*P* > 0.05).

### 3.4. Fetal MCA BFPs before and after Treatment

Color Doppler ultrasound based on denoising algorithm (Table 4) showed that there was no great difference between the two groups of fetal PI, RI, S/D, and PSV before treatment (*P* > 0.05); after treatment, the PI, RI, and S/D in group A were much lower than the above indicators in group B (*P* < 0.05), but there was no marked difference in the PSV between two groups (*P* > 0.05).

### 3.5. Fetal CPR before and after Treatment

CPR referred to the ratio of MCA PI to UA PI. The CPR was not statistically and greatly different between the two groups before treatment (*P* > 0.05), and the CPR in group A was lower obviously than that in group B (*P* < 0.05), as given in Table 5.

### 3.6. Fetal Growth Index

Color Doppler ultrasound based on the denoising algorithm showed that the growth indicators of fetuses in group A were markedly better, and the differences between the groups were obvious statistically (*P* < 0.05) (Table 6).

### 3.7. Maternal and Child Outcome in Two Groups

As shown in Tables 7 and 8, there was no great difference between the two groups in terms of maternal and infant adverse events (*P* > 0.05), but the Apgar score, weight, and gestational age of newborns in group A were obviously higher than those in group B (*P* < 0.05).

### 3.8. Image Comparison before and after LPG-PCA Denoising

A 31-year-old woman was initially screened for FGR two weeks ago. When the diagnosis was further confirmed, the image quality was not high due to redundant interference noise in the Doppler ultrasound image, which affected the diagnosis of the condition. After the optimization of the LPG-PCA algorithm, the noise was effectively removed, and the image clarity was improved (Figure 2).

## 4. Discussion

LMWH has the characteristics of easy absorption, quick onset, and few adverse reactions [12]. It will not pass through the placental barrier, so it is safe and effective to treat FGR, improve antithrombin III activity and blood hypercoagulability, and ensure the integrity of vascular endothelium, so as to protect the function of vascular endothelial cells [13,14]. In addition, the drug also has anti-inflammatory and lipid-regulating effects, accelerates the blood supply of pregnant women, and promotes fetal growth by regulating the intrauterine microenvironment [15,16]. As an antiplatelet aggregation drug, aspirin can accelerate blood circulation and increase the flow of blood between the placenta and the fetus, thereby improving the fetal nutrition supply [17,18]. The combination of the two can ensure that the placenta gets adequate nutrition and maintain normal pregnancy.

Color Doppler ultrasound is an ultrasound diagnostic technology that uses color images to display the direction and relative velocity of blood flow in real time on the basis of two-dimensional gray-scale ultrasound images. It is the most accurate and most widely used ultrasound examination method, and its judgment and sensitivity of the nature of the disease is much higher than that of ordinary examination [19]. However, due to imaging equipment and other reasons, unnecessary interference information such as noise often appears in color Doppler ultrasound images, which affects the image quality and makes the readers unable to make accurate judgments of the disease, causing troubles in clinical work. Therefore, the LPG-PCA denoising algorithm was applied to color Doppler ultrasound technology in this study, which can effectively remove noise, clearly display, and improve imaging accuracy. It was applied in 40 cases of group B pregnant women who were treated with LMWH calcium injection and 40 cases of pregnant women in group A who were treated with aspirin enteric-coated tablets. The imaging results showed that the total effective rate in group A (87.5%) was obviously higher than that of group B (62.5%), and the difference was statistically significant (*P* < 0.05), indicating that the combined scheme can further improve the prognosis. After treatment, the PI (0.72 ± 0.19), RI (0.57 ± 0.17), and S/D (2.26 ± 0.43) in group A were much lower than the previously mentioned indicators in group B, which were 0.92 ± 0.21, 0.75 ± 0.14, and 2.64 ± 0.45, respectively (*P* < 0.05). AFI (13.71 ± 2.2) was much higher than group B (11.38 ± 2.16) (*P* < 0.05), indicating that combined therapy can better improve the blood perfusion state of the fetus and the quality of amniotic fluid. The growth indicators of fetuses in group A were much better (*P* < 0.05) in contrast to those in group B. There was no notable difference in adverse events between the two groups of mothers and infants (*P* > 0.05), but the Apgar score, weight, and gestational age of newborns in group A were all greatly higher than those in group B (*P* < 0.05). Such results showed that the addition of aspirin treatment would not increase the adverse events of the mother and the baby, but it can promote the development of the fetus with good safety.

## 5. Conclusion

In this study, 80 FGR pregnant women were grouped into an experimental group (aspirin enteric-coated tablets + LMWH calcium injection) and a control group (LMWH calcium injection) according to the different treatment plans, with 40 cases in each group. All patients underwent Dopper ultrasound imaging. A two-stage image denoising by principal component analysis (PCA) with local pixel grouping (LPG-PCA) denoising algorithm was constructed for enhancement process of Ultrasound images. The BFPs, MCA BFPs, CPR, AFI, and PO of the two groups were compared. The results suggested that the combined treatment of FGR with aspirin and LMWH, compared with single LMWH treatment, can not only improve the clinical effect, but also better improve the hemodynamic parameters and amniotic fluid quality of the child and promote fetal growth. In addition, it would not greatly increase the adverse maternal and infant outcome, so it was clinically suitable for promotion. However, the sample size of pregnant women selected in this study was small and the source was single, which may affect the accuracy of the results. Later, it will consider collecting more patient cases to further explore the application value of ultrasound imaging based on artificial intelligence algorithms in clinical diagnosis.

## Figures and Tables

**Figure 1:** Specific flowchart of the algorithm.

**Figure 2:** Image comparison before and after LPG-PCA denoising. (a) The original ultrasound image; (b) the ultrasound image obtained after denoising.

**Table 1:** Basic data of patients.

Group	Age (years)	BMI (kg/m^2^)	Average gestational week at admission (weeks)	Menstrual women/primiparous women (cases)
Group A	31.73 ± 7.05	24.56 ± 1.28	35.06 ± 3.15	21/19
Group B	32.34 ± 7.63	24.37 ± 1.37	35.12 ± 3.08	18/22

BMI: body mass index.

**Table 2:** Comparison on clinical efficacy.

Group	Markedly effective	Effective	Ineffective	Total effective rate (%)
Group A	21	14	5	87.5
Group B	12	13	15	62.5

**Table 3:** Comparison of fetal UA BFPs and AFI before and after treatment.

Group	Group A		Group B	
	Before treatment	After treatment	Before treatment	After treatment
PI	1.29 ± 0.26	0.72 ± 0.19^#∗^	1.28 ± 0.29	0.92 ± 0.21^#∗^
RI	1.00 ± 0.18	0.57 ± 0.17^#∗^	1.02 ± 0.19	0.75 ± 0.14^#∗^
S/D	3.20 ± 0.41	2.26 ± 0.43^#∗^	3.18 ± 0.52	2.64 ± 0.45^#∗^
PSV (s)	50.42 ± 10.08	41.6 ± 10.13	52.01 ± 11.14	42.87 ± 11.39
AFI (cm)	10.28 ± 1.96	13.71 ± 2.21	10.36 ± 2.07	11.38 ± 2.16

*Note.* # suggests that the difference was statistically obvious compared with the value before treatment in the same group (*P* < 0.05), and  ^*∗*^ indicates that the difference was statistically great in contrast to the value in group B (*P* < 0.05).

**Table 4:** Comparison on fetal MCA BFPs and AFI before and after treatment.

Group	Group A		Group B	
	Before treatment	After treatment	Before treatment	After treatment
PI	1.78 ± 0.26	1.31 ± 0.18^#^ ^*∗*^	1.75 ± 0.23	1.73 ± 0.25^#∗^
RI	1.23 ± 0.05	0.75 ± 0.03^#^ ^*∗*^	1.26 ± 0.04	0.81 ± 0.05^#∗^
S/D	5.38 ± 0.61	3.75 ± 0.58^#^ ^*∗*^	5.45 ± 0.64	5.11 ± 1.09^#∗^
PSV	50.03 ± 12.86	42.01 ± 13.86	50.15 ± 13.82	43.52 ± 13.51

*Note.* # suggests that the difference was statistically obvious compared with the value before treatment in the same group (*P* < 0.05), and  ^*∗*^ indicates that the difference was statistically great in contrast to the value in group B (*P* < 0.05).

**Table 5:** Comparison of fetal CPR in two groups before and after treatment.

Group	Group A		Group B	
	Before treatment	After treatment	Before treatment	After treatment
CPR	1.379	1.81^#∗^	1.367	1.88^#∗^

*Note.* # suggests that the difference was statistically obvious compared with the value before treatment in the same group (*P* < 0.05), and  ^*∗*^ indicates that the difference was statistically great in contrast to the value in group B (*P* < 0.05).

**Table 6:** Average weekly fetal growth indicators for the two groups.

Group	Fetal double parietal diameter (mm)	Femur diameter (mm)	Head circumference (cm)	Abdominal circumference (cm)	Uterine height (cm)
Group A	2.4 ± 0.9^∗^	2.2 ± 0.6^∗^	1.2 ± 0.4^∗^	1.3 ± 0.7^∗^	0.8 ± 0.3^∗^
Group B	1.8 ± 0.4	1.7 ± 0.5	0.8 ± 0.2	0.9 ± 0.4	0.4 ± 0.6

*Note.* ^*∗*^ indicates that the difference was statistically great in contrast to the value in group B (*P* < 0.05).

**Table 7:** Comparison of adverse events between the two groups.

Group	Placental abruption	Fetal distress	Oligohydramnios	Postpartum hemorrhage
Group A	1	1	2	2
Group B	2	1	1	2

**Table 8:** Comparison of neonatal outcomes between the two groups.

Group	Apgar score	Weight (kg)	Gestational age (weeks)	Choking	Premature delivery	Very low weight	Full-term infants
Group A	9.17 ± 0.26 ^*∗*^	3.57 ± 1.08 ^*∗*^	38.85 ± 2.50 ^*∗*^	1	0	0	1
Group B	7.33 ± 0.25	2.61 ± 1.13	36.18 ± 2.25	1	1	1	2

*Note.* ^*∗*^ indicates that the difference was statistically great in contrast to the value in group B (*P* < 0.05).

## Data Availability

The data used to support the findings of this study are available from the corresponding author upon request.
